The article "Study on the Efficacy and Safety of Ambroxol Combined with Methylprednisolone in Patients with Acute Lung Injury" was retracted in 2024. Reasons: signs of a paper mill; suspected computer-generated content; unreliable results or conclusions; concerns about the data.

# Study on the Efficacy and Safety of Ambroxol Combined with Methylprednisolone in Patients with Acute Lung Injury

**DOI:** 10.1155/2021/5771101

**Published:** 2021-11-28

**Authors:** Weiwei Su, Qinglian Dong, Fangfang Jiao

**Affiliations:** Department of Critical Care Medicine, Dongying People's Hospital of Shandong Provincial Hospital Group, Dongying, Shandong Provincial, China

## Abstract

**Background:**

There is no better treatment method towards paraquat-induced acute lung injury (ALI) at present. Ambroxol combined with methylprednisolone exhibits a significant improvement effect on ALI treatment, whereas their mechanism in ALI is still unclear.

**Methods:**

64 patients with ALI caused by paraquat poisoning brought to our hospital from January 2015 to January 2018 were selected. They were separated into a combined treatment group (CTG) and a routine treatment group (RTG) on the basis of different treatment methods. The survival of patients was observed after 7 days of treatment. Arterial blood gas, oxygen partial pressure (PaO_2_), partial pressure of carbon dioxide (PaCO_2_), oxygenation index (PaO_2_/FiO_2_), patient's spontaneous respiratory rate (RR), tidal volume (VT), and positive end-expiratory pressure (PEEP) were observed before and after treatment for 7 days. Interleukin 6 (IL-6) and tumor necrosis factor *α* (TNF-*α*) were analyzed. The differences of indexes between the dead patients and the survivors were observed, and the potential predictive value of death was analyzed.

**Results:**

After treatment, the indexes of patients were significantly improved in both groups compared with those before therapy. Further comparison showed that the improvement of PaO_2_, PaCO_2_, and PaO_2_/FiO_2_ in CTG was obviously higher than that in RTG (*p* < 0.05). The improvement of RR, PEEP, and VT in CTG was obviously higher than that in RTG (*p* < 0.05). The decreased degree of IL-6 and TNF-*α* in CTG was higher than that in RTG (*p* < 0.05). The 7-day mortality rate of 64 patients was 39.06%, and there was no obvious difference in the 7-day survival rate in both groups (*p* = 0.649). IL-6 and TNF-*α* were expected to be potential prediction indexes of paraquat-induced ALI.

**Conclusion:**

Ambroxol combined with methylprednisolone significantly improved the oxygen partial pressure and oxygenation index of patients with paraquat-induced ALI and inhibited the inflammatory response of patients.

## 1. Introduction

Paraquat belongs to bipyridyliums. Because of its broad-spectrum activity, high-efficiency, limited environmental pollution, and ease of use, it is widely applied in agriculture production all over the world, especially in developing countries [1]. However, it is also highly toxic to human beings and animals, mainly because its redox activity generates reactive oxygen species (ROS) [2]. Although paraquat is extremely toxic to human beings and livestock at present, there is no specific toxinicide [3].

After paraquat poisoning, it accumulates in human lungs and is prone to acute lung injury (ALI) and pulmonary fibrosis [4, 5]. Currently, a patient is mainly treated clinically by dialysis combined with drug therapy after paraquat poisoning [6]. Ambroxol is a new mucolytic agent. In recent years, many reports reveal that ambroxol plays a vital role in protecting the respiratory system [7]. Methylprednisolone has strong anti-inflammatory and anti-immune effects. Early application of methylprednisolone can improve the body's tolerance to harmful factors, reduce severe inflammatory reaction caused by paraquat poisoning, reduce inflammatory exudation, and has an antifibrosis effect [8, 9]. Previous studies have found that [10] high-dose ambroxol has an objective effect in the treatment of ALI caused by paraquat poisoning. However, there are few studies on the treatment of paraquat-induced ALI by high-dose ambroxol combined with methylprednisolone. It is not clear whether large doses of combined drugs can improve the patient's disease.

Therefore, this research was aimed at exploring the effect of high-dose ambroxol combined with methylprednisolone on the improvement of patients with ALI caused by paraquat and its influence on survival, hoping to furnish reference for clinical treatment.

## 2. Methods and Data

### 2.1. Clinical Data

From January 2015 to January 2018, 64 patients with ALI caused by paraquat poisoning brought to our hospital were selected, including 48 men and 16 women, with an average age of 35.6 ± 8.4 years old. Patients were separated into a high-dose treatment group (*n* = 34) and RTG (*n* = 30) on the basis of different treatment schemes.

Inclusion criteria were as follows: all patients were poisoned by paraquat and did not take other pesticides. The patients were confirmed to have ALI within 0-6 hours after taking paraquat during admission, and their families signed informed consent.Exclusion criteria were as follows: comorbid with tumor, cardiovascular, and cerebrovascular diseases; patients who died within 1 day after admission.

This research was ratified by the Medical Ethics Committee of our hospital.

### 2.2. Methods of Treatment

In this research, patients underwent gastric lavage and catharsis first in the two groups, and then, hemoperfusion and hemodialysis were used to treat patients for 4~6 h, once/d, for 3~4 d in succession. In addition, the patients were ventilated by ventilator (SIMV+PsV+PEEP mode). In RTG, the patients were injected intravenously with 500 mg/d methylprednisolone for 3 days, followed by a dose reduction. It was supplemented by antioxidation, liver protection, myocardial nutrition, maintenance of water electrolyte, acid-base balance, etc. On this basis, patients in CTG were given 20 mg/kg/d ambroxol hydrochloride injection by intravenous infusion for 12 h for 3-5 days.

### 2.3. ELISA Test

The expressions of IL-6 and TNF-*α* were detected through ELISA (Shanghai Enzyme-Linked Biotechnology Co., Ltd., PI330, PT518). The blank hole, standard sample hole, and sample hole to be tested were set up. 50 *μ*L of standard product was added into the standard sample hole with different concentrations. The 10 *μ*L sample to be tested was first put in the sample well, and then, the 40 *μ*L sample diluent was added. Nothing was added to the blank well. In addition to the blank well, 100 *μ*L of HRP-labeled detection antibody was put in each of the standard hole and the sample hole. The reaction holes were sealed with a sealing plate membrane and cultivated in a water bath at 37°C for 65 min. The liquid was discarded, and absorbent paper was used to pat dry. Each hole was filled with washing liquid and allowed to stand for 2 min, the washing liquid was thrown out, and absorbent paper was used to pat dry. This was repeated 6 times. Each 50 *μ*L of substrates A and B was put in each hole and cultivated at 37°C in the dark for 10 min. The 50 *μ*L of terminal liquid was added to each hole, and OD values of each hole were tested at the wavelength of 450 nm within 15 min to calculate the concentration.

### 2.4. Outcome Measures

Main outcome measures were as follows: to observe the survival of patients after 7 days of treatment; to observe the arterial blood gas, PaO_2_, PaCO_2_, and oxygenation index (PaO_2_/FiO_2_) before and after treatment for 7 days; to observe the spontaneous RR, VT, and PEEP before and after treatment for 7 days; and to observe the IL-6 and TNF-*α* before and after treatment for 7 days.

The secondary observation index is as follows: to compare the baseline data of patients in the two groups and to observe the differences of various indexes between the dead patients and the survivors and analyze the potential predictive value of death.

### 2.5. Statistical Analysis

In this research, SPSS20.0 was applied to make statistical analysis on the collected data, and GraphPad 7 was applied to draw the required pictures. The general data of patients were analyzed by the chi-square test. The biological indexes of patients were analyzed by *t*-test, in which the normal distribution data was represented by mean number ± standard deviation (mean ± SD). The independent sample *t*-test was used for intergroup comparisons. The data that did not accord with the normal distribution was represented by quartile. ROC was applied to plot the potential predicting value of each index of dead patients and survivors. K-M survival curve was applied to analyze the 7-day survival of patients in the two groups. *p* < 0.05 indicated that there was statistical difference.

## 3. Results

### 3.1. Comparison of Baseline Data

In this study, we first compared the baseline data of patients in RTG and CTG. Through analysis, we found that there were no statistical differences in the age, gender, BMI (body mass index), history of smoking, place of residence, educational level, and LIS score in both groups (*p* > 0.05) (Table 1).

### 3.2. Changes of Blood Gas Indexes before and after Treatment

In this study, the changes of blood gas indexes were compared in both groups before and after treatment. By comparing, we found that there was no significant difference in PaO_2_, PaCO_2_, and PaO_2_/FiO_2_ in both groups before therapy (*p* > 0.05). Further comparing the changes before and after treatment, we found that PaO_2_, PaCO_2_, and PaO_2_/FiO_2_ increased significantly in both groups after therapy (*p* < 0.01). By further comparing, we found that the improvement of PaO_2_, PaCO_2_, and PaO_2_/FiO_2_ in CTG was obviously higher than that in RTG (*p* < 0.05) (Figure 1).

### 3.3. Changes of Respiratory Parameters before and after Treatment

In this study, the changes of respiratory parameters were compared in both groups before and after treatment. By comparing, we found that there was no obvious difference in RR, PEEP, and VT in both groups before treatment (*p* > 0.05). Further comparing the changes before and after treatment, we found that RR and PEEP reduced obviously in the two groups after therapy (*p* < 0.01), while VT increased significantly. By further comparing, we found that the improvement of RR, PEEP, and VT in CTG was obviously higher than that in RTG (*p* < 0.05) (Figure 2).

### 3.4. Changes of Inflammatory Factors before and after Treatment

In addition, we also detected the levels of IL-6 and TNF-*α* in patients' serum before and after therapy. Through comparison, we found that there were no statistical differences in the levels of IL-6 and TNF-*α* in patients' serum before treatment (*p* > 0.05), while after therapy, the levels of IL-6 and TNF-*α* in patients' serum were obviously lower than before treatment (*p* < 0.01). Further analysis, we found that the decreasing degrees of IL-6 and TNF-*α* of patients in CTG were higher than those in RTG (*p* < 0.05) (Figure 3).

### 3.5. Survival of Patients

We have made statistics on the 7-day survival of patients. The 7-day mortality rate of 64 patients was 39.06%. Based on further analysis of the survival in the two groups, it showed that the mortality rate of patients in RTG was 40.00% and that in CTG was 38.23%. There were no statistical differences in the 7-day survival rate in both groups (*p* = 0.649) (Figure 4).

### 3.6. Predictive Value of Each Index on the Death of Patients before Treatment

At the end of the study, we analyzed the value of each index in predicting the death of patients, and patients were separated into the death group (*n* = 25) and the survival group (*n* = 39) on the basis of the death situation of patients. The changes of blood gas index, respiratory parameters, and inflammatory factors were further compared before treatment. Through analysis, we found that there was no statistical difference in PaCO_2_, PaO_2_/FiO_2_, RR, PEEP, and VT of patients between the death group and the survival group (*p* > 0.05). PaO_2_ in the death group was obviously lower than that in the survival group, and IL-6 and TNF-*α* in the death group were obviously higher than those in the survival group, and there was statistical difference (*p* < 0.05). Then, we drew an ROC curve according to the different indexes. The results showed that the area under the PaO_2_ curve was 0.641, the area under the IL-6 curve was 0.757, and the area under the TNF-*α* curve was 0.701. Among them, IL-6 and TNF-*α* were expected to be potential prediction indexes of ALI caused by paraquat (Figures 5 and 6 and Table 2).

## 4. Discussion

Paraquat is a common herbicide in developing countries due to its remarkable herbicidal effect and low cost [11]. At present, the main treatment schemes for paraquat poisoning clinically include gastric lavage, catharsis, activated carbon adsorption, hemoperfusion, antioxidant free radical drugs, and immunosuppressive agents [12–14]. Although the survival time of the patients is prolonged, the prognosis of the patients is still not significantly improved. The main cause of death is ALI [15]. In this study, we found that ambroxol combined with methylprednisolone had improved the inflammatory response and disease condition in patients with paraquat-induced ALI. We also found that IL-6 and TNF-*α* had high clinical value in predicting the 7-day survival of patients and were expected to become potential clinical predictors.

In this study, we found that ambroxol combined with methylprednisolone on the basis of conventional treatment significantly improved the oxygen partial pressure and oxygenation index of patients, suggesting that combined medication might improve pulmonary hyperemia/exudation, regulate lung compliance, and inhibit the development of ALI. Ambroxol, as a mucus drainage promoter, can cleave acidic mucopolysaccharide fibers in sputum, inhibit the synthesis process of acidic mucopolysaccharide fibers in goblet cells and glands, form obvious stimulation to mucous cells, enhance adhesion of small molecules of mucus, and increase protein secretion, thereby reducing mucus and sputum viscosity, realizing effective sputum dilution, reducing sputum cough difficulty, reducing incidence of cilia adhesion, and further improving the respiratory condition of patients [16, 17]. Methylprednisolone, as a glucocorticoid, has rapid onset and anti-inflammatory effects in the treatment of ALI, and it has therapeutic effects on many links of inflammatory reaction. In addition, it can increase local blood flow and inhibit the release of the proteolytic enzyme [18, 19]. The combined use of the two drugs further improved the patient's inflammatory reaction and increased the patient's oxygen partial pressure and oxygenation index.

Previous reports have shown that [20] ambroxol alleviates ventilator-induced lung injury by inhibiting c-Jun, and it also plays an inhibitory role on the occurrence of inflammatory reactions in the body of patients. In the studies of Theroux et al. [21], it has shown that preventive methylprednisolone can reduce inflammation in children and improve the result of one-time lung ventilation. In our study, it was found that the expression of IL-6 and TNF-*α* in patients' peripheral venous blood was further reduced after the combination of drugs, suggesting that the combination of drugs reduced the inflammatory reaction of patients, which was similar to the results of the above study. It also suggested that ambroxol combined with methylprednisolone played a positive effect in improving ALI caused by paraquat.

At the end of the research, we made a short-term observation on the survival of the patients, and it was found that the two treatment schemes had no obvious influence on the patients' 7-day survival. In addition, patients were further separated into groups on the basis of their survival conditions. To observe the connection of various indexes with the patients' survival, the results showed that PaO_2_ in the dead group was obviously lower than that in the survival group, while the expression of IL-6 and TNF-*α* in the dead group was higher than that in the survival group. Then, we further drew an ROC curve and found that IL-6 and TNF-*α* had higher clinical value in calculating the patients' short-term survival. However, we still need to further explore its potential mechanism.

There are still some limitations in this study. First of all, we have not conducted a long-term follow-up survey on patients. In addition, due to the small sample size, deviation may be caused to the data results. Therefore, we hope to increase our sample size in future studies and conduct long-term follow-up of patients, so as to supplement our research conclusions. Different doses of ambroxol might have negative effects on host defenses. Therefore, more work will be necessary in clinics to find an optimal therapeutic dosage of ambroxol with minimal side effects.

To sum up, ambroxol combined with methylprednisolone significantly improved the oxygen partial pressure and oxygenation index of patients with paraquat-induced ALI and inhibited the inflammatory response of patients.

## Figures and Tables

**Figure 1:** Changes of blood gas indexes before and after treatment. (a) Changes of PaO_2_ before and after treatment were detected by blood gas analysis. (b) Changes of PaCO_2_ before and after treatment were detected by blood gas analysis. (c) Changes of PaO_2_/FiO_2_ before and after treatment were detected by blood gas analysis. ^∗^*p* < 0.05 and ^∗∗^*p* < 0.01.

**Figure 2:** Changes of respiratory parameters before and after treatment. (a) Analysis on the changes of RR before and after treatment. (b) Analysis on the changes of PEEP before and after treatment. (c) Analysis on the changes of VT before and after treatment. ^∗^*p* < 0.05 and ^∗∗^*p* < 0.01.

**Figure 3:** Changes of IL-6 and TNF-*α* before and after treatment. (a) ELISA was used to detect changes of IL-6 before and after treatment. (b) ELISA was used to detect the changes of TNF-*α* before and after treatment. ^∗^*p* < 0.05 and ^∗∗^*p* < 0.01.

**Figure 4:** Effect of different treatment methods on patients' 7-day survival.

**Figure 5:** Expressions of blood gas index, respiratory parameters, and inflammatory factor before treatment in patients with death and survival. (a) PaO_2_ expression before treatment in patients with death and survival. (b) PaCO_2_ expression before treatment in patients with death and survival. (c) PaO_2_/FiO_2_ expression before treatment in patients with death and survival. (d) RR expression before treatment in patients with death and survival. (e) PEEP expression before treatment in patients with death and survival. (f) VT expression before treatment in patients with death and survival. (g) IL-6 expression before treatment in patients with death and survival. (h) TNF-*α* expression before treatment in patients with death and survival.

**Figure 6:** ROC curve area of PaO_2_, IL-6, and TNF-*α*. (a) PaO_2_ was used to predict the area under the curve of paraquat-induced ALI. (b) IL-6 was used to predict the area under the curve of paraquat-induced ALI. (c) TNF-*α* was used to predict the area under the curve of paraquat-induced ALI.

**Table 1:** Comparison of baseline data.

Factors		RTG (*n* = 34)	CTG (*n* = 30)	*p* value
Age				0.679
	≥35 years old (*n* = 38)	21	17	
	<35 years old (*n* = 26)	13	13	
Gender				0.148
	Male (*n* = 48)	28	20	
	Female (*n* = 16)	6	10	
BMI (kg/m^2^)		22.41 ± 1.82	21.94 ± 1.58	0.277
Smoking history				0.251
	Yes (*n* = 45)	26	19	
	No (*n* = 19)	8	11	
Place of residence				0.839
	City (*n* = 20)	11	9	
	Rural (*n* = 44)	23	21	
Educational level				0.765
	≥Junior high school (*n* = 29)	16	13	
	<Junior high school (*n* = 35)	18	17	
LIS score		2.15 ± 0.48	2.10 ± 0.58	0.707

**Table 2:** ROC parameters of PaO_2_, IL-6, and TNF-*α*.

Indicators	AUC	*p* value	Specificity	Sensitivity	Youden index	Cut-off
PaO_2_	0.641	0.059	100.00%	33.33%	33.33%	>50.52
IL-6	0.757	0.001	100.00%	46.15%	46.15%	<43.67
TNF-*α*	0.701	0.007	88.00%	48.71%	36.72%	<182.11

## Data Availability

The authors confirm that the data supporting the findings of this study are available within the article.

## References

[1] Kumar T. S., Ranjan M. R., Smita D. (2019). Paraquat poisoning. *The Journal of the Association of Physicians of India*.

[2] Sun B., He Y. (2017). Paraquat poisoning mechanism and its clinical treatment progress. *Zhonghua Wei Zhong Bing Ji Jiu Yi Xue*.

[3] Dinis-Oliveira R. J., Duarte J. A., Sanchez-Navarro A., Remiao F., Bastos M. L., Carvalho F. (2008). Paraquat poisonings: mechanisms of lung toxicity, clinical features, and treatment. *Critical Reviews in Toxicology*.

[4] Zhang F., Hu L., Wu Y. X. (2019). Doxycycline alleviates paraquat-induced acute lung injury by inhibiting neutrophil-derived matrix metalloproteinase 9. *International Immunopharmacology*.

[5] Zhang L., Li Q., Liu W., Liu Z., Shen H., Zhao M. (2019). Mesenchymal stem cells alleviate acute lung injury and inflammatory responses induced by paraquat poisoning. *Medical Science Monitor*.

[6] Shen H., Wu N., Wang Y. (2017). Chloroquine attenuates paraquat-induced lung injury in mice by altering inflammation, oxidative stress and fibrosis. *International Immunopharmacology*.

[7] Cazan D., Klimek L., Sperl A., Plomer M., Kolsch S. (2018). Safety of ambroxol in the treatment of airway diseases in adult patients. *Expert Opinion on Drug Safety*.

[8] Tu G. W., Shi Y., Zheng Y. J. (2017). Glucocorticoid attenuates acute lung injury through induction of type 2 macrophage. *Journal of Translational Medicine*.

[9] Zhang G., Zhang X., Huang H., Ji Y., Li D., Jiang W. (2018). Saquinavir plus methylprednisolone ameliorates experimental acute lung injury. *Brazilian Journal of Medical and Biological Research*.

[10] Wu X., Li S., Zhang J. (2014). Meta-analysis of high doses of ambroxol treatment for acute lung injury/acute respiratory distress syndrome based on randomized controlled trials. *The Journal of Clinical Pharmacology*.

[11] Kumar S. (2016). Paraquat tongue. *Indian Journal of Gastroenterology*.

[12] de Pont A., Volbeda M. (2018). Extracorporeal treatment for paraquat poisoning. *Critical Care Medicine*.

[13] Dorooshi G., Zolfaghari S., Eizadi-Mood N., Gheshlaghi F. (2018). A new treatment approach for acute paraquat poisoning. *Journal of Research in Pharmacy Practice*.

[14] Oghabian Z., Williams J., Mohajeri M. (2019). Clinical features, treatment, prognosis, and mortality in paraquat poisonings: a hospital-based study in Iran. *Journal of Research in Pharmacy Practice*.

[15] Jiang C., Zhong R., Zhang J. (2019). Reduning injection ameliorates paraquat-induced acute lung injury by regulating AMPK/MAPK/NF‐*κ*B signaling. *Journal of cellular biochemistry*.

[16] Ge L. T., Liu Y. N., Lin X. X. (2016). Inhalation of ambroxol inhibits cigarette smoke-induced acute lung injury in a mouse model by inhibiting the Erk pathway. *International Immunopharmacology*.

[17] Zhang S. J., Jiang J. X., Ren Q. Q. (2016). Ambroxol inhalation ameliorates LPS-induced airway inflammation and mucus secretion through the extracellular signal-regulated kinase 1/2 signaling pathway. *European Journal of Pharmacology*.

[18] Feng S. Y., Gao J., Wang J., Li Y. (2018). Effects of prolonged methylprednisolone treatment after pulse therapy for paraquat-intoxicated rats. *Human & Experimental Toxicology*.

[19] Ji Y., Zhang G., Zhu H., Li D., Jiang W. (2018). Indinavir plus methylprednisolone ameliorates experimental acute lung injury in vitro and in vivo. *Shock*.

[20] Cao D. W., Hou M. X., Zhang X. R. (2019). Ambroxol alleviates ventilator-induced lung injury by inhibiting c-Jun expression. *Eur Rev Med Pharmacol Sci*.

[21] Theroux M. C., Fisher A. O., Rodriguez M. E. (2015). Prophylactic methylprednisolone to reduce inflammation and improve outcomes from one lung ventilation in children: a randomized clinical trial. *Pediatric Anesthesia*.

